This article has been retracted.

# The relationship between political instability and stock market performance: An analysis of the MSCI index in the case of Pakistan

**DOI:** 10.1371/journal.pone.0292284

**Published:** 2023-10-19

**Authors:** Zhiying Mai, Hassan Mujtaba Nawaz Saleem, Muhammad Kamran

**Affiliations:** 1 International Business College, Shaanxi Normal University, Xi’An, Shaanxi Province, China; 2 Department of Management Sciences, The Islamia University of Bahawalpur, Punjab, Pakistan; 3 MNS University of Engineering and Technology Multan, Punjab, Pakistan; University of City Island, CYPRUS

## Abstract

The stock market is the barometer of the economy that reflects the overall health and direction of the economic development and is affected by different factors including social, environmental and political. It is important to investigate the effect of the political instability on the stock market performance, especially on emerging economies. Therefore, we aim to study the relationship between political instability and stock market performance in Pakistan. To meet our objectives, we used past data from 1996 to 2021. Data are collected from the DataStream data base. MSCI indices are used as the proxy for the Stock market performance of the selected country. World governance six indicators are used in the study as the explanatory variable concentrating the political instability index as the main explanatory variable. Regression analysis is used but two-way robustness analysis was done for the accuracy of the findings through GMM methods and taking GDP as another endogenous variable. Our findings shows that the political stability has significant positive impact on the stock market performance while, political instability has negative impact on stock market performance. Moreover, other governance indicators has a significant positive impact on performance. However, political instability disrupts the operations and economical activities that leads to decrease the investor confidence and also decrease the foreign investment with the increment of the risk in the country. Moreover, our study has some implications for investors to develop the diversified portfolio to minimize the risk and policy makers can increase their foreign direct investment within the economy by controlling the political instability.

## 1. Introduction

The stock market is the backbone of economy that provides to the direction of the growth towards achieving the economic goal but in that way, there is many obstacles that faced by the stock market such as political instability in shape strikes, lack of proper decision and the code of corruptions. Many other social as well as economic factors also affect the stock market performance. We investigated the political instability effect on stock market performance especially in Pakistan on the ground Pakistan faced higher political instability from last two decades and its intensity increasing day by days. Therefore, the relationship between political instability and market performance is a complex issue, and it varies significantly depending on the country and the specific political situation. Political instability had a significant impact on a country’s economy. Political instability led to uncertainty, lack of investment, and a decrease in economic growth.

There are limited studies on the relationship between political instability and the stock market performance in the emerging economies, to address this type of the literature we selected the Pakistan an emerging economy for the investigation because Pakistan was affected from the political instability since independence. Moreover, governance mechanism of any economy has the significant for the development that is limited discussion in the previous body of the literature on country governance mechanism that affect the stock market. Moreover, previous studies investigate the relationship between these variables by using different methods, but this study fulfill the gap by investigating two effective methodology regression analysis and the GMM method for robustness analysis.

We aim to fill the gap with three objectives, first is to investigate the relationship between the political instability and the stock market performance in Pakistan. Second, is to investigate the relationship between governance indicators (such as control of corruption, voice and accountability, regulatory quality, rules of law, government effectiveness) and stock market performance. Third objectives include, is to investigate the change in the performance by taking robustness of the endogenous variable MSCI index to gross domestic product (GDP) growth rate for the accuracy of the findings that provide another novelty to the research.

Our study contributed to the existing body of knowledge in the following ways. First, it contributes to fresh evidence in the empirical and theoretical literature in context of the emerging economy Pakistan. Secondly, it contributes to literature that the not only the political instability decrease the stock market performance but also the lower control of corruption also other consequences in damaging the stock market reputation that decrease the investor confidence on the market. The voice and accountability also increase the stock market performance but in this way we added in the literature of the [1] that free media and accountability leads to rise in the stock prices but some studies have argued that media bias and sensationalism in reporting lead to misinterpretations or exaggerations of market events, which might increase market volatility and lead to short-term fluctuations. However, the regulatory quality and the rules of law in the economy leads to rise the stock prices that shows the government effectiveness in term of policy implementation and the code of conduct and governance control, and these points make another significant contribution in the existing literature by this study. Moreover, our study contributed by providing the significant implications for the investors, government and the policy makers. Based on the findings of this study, governments take measures to address political instability and establish a stable political environment. This can be achieved through policies that promote political stability, like constitutional reforms, and by addressing the root causes of political instability, such as poverty and inequality. By using the findings of the research, the governments and the policy makers can improve transparency and accountability in the political system to boost investor confidence.

The rest of the article is organized in the following manner. Part 2 provides an overview of recent literature and theoretical background and proposes several hypotheses that can be tested to elucidate the relationship between variables. The conceptual framework, research design, and methods are outlined in Part 3. Section 4 presents the study’s findings, while Section 5 includes the conclusion, suggestions for further research, limitations, and practical implications.

## 2. Literature review

There have been several studies that have examined the impact of political instability on the economy through the use of MSCI index values. [2] found that political instability in emerging markets has a significant negative impact on stock market performance as measured by the MSCI Emerging Markets Index. The study found that political instability was negatively correlated with MSCI index values, and that this relationship was stronger in more developed countries. However, this study did not use Political Instability Index for selecting the political crises affecting the selected countries that is the gap in the existing literature related to emerging economies but this gap is filled by using the world governance indicator political stability within Pakistan. [3] found that political instability in emerging markets has a significant negative impact on the performance of the MSCI Emerging Markets Index and also found that political instability was negatively correlated with MSCI index values, and again that this relationship was stronger in more developed countries. [4] found that political instability in emerging markets has a significant negative impact on the performance of the MSCI Emerging Markets Index. The study found that political instability was negatively correlated with MSCI index values, and that this relationship was stronger in more developed countries. Similarly, [5] also found that political instability had a greater negative impact on the MSCI Emerging Markets Index than on the MSCI World Index.

[6] found that the political factor influences the stock market that leads to uncertainty and lack of confidence by the investors which decrease the stock market prices in Pakistan. In 2018 Pakistan experienced a period of political instability due to the general elections and subsequent disputes over the election results. During this time, the Karachi Stock Exchange (KSE) saw a decline in its performance. Similarly, in 2020, when the COVID-19 pandemic hit Pakistan, it led to political instability as well as economic uncertainty. This caused a drop in the KSE-100 Index, which is the benchmark index of the Pakistan Stock Exchange [7]. Moreover, there have been several studies that have investigated the relationship between political instability and stock market performance in emerging economies. One study by [8] examined the impact of political instability on stock market returns from 2000 to 2014 and found that political instability had a significant negative impact on stock market returns, particularly in the short run, and also suggest that political instability can create uncertainty and reduce investor confidence, leading to a decline in stock market returns.

Another study by [9] investigated the impact of political instability on stock market volatility from 1992 to 2015 and found that political instability had a significant positive impact on stock market volatility, indicating that political instability lead to higher levels of risk and uncertainty in the stock market. A study by [10] analyzed the impact of political instability and macroeconomic factors on stock market performance from 2002 to 2019 and found that political instability had a negative impact on stock market returns, but the effect was less significant when controlling for other macroeconomic factors such as interest rates and inflation.

A study by [11] found that political instability can lead to lower economic growth and investment in developing countries, including Pakistan. A study by [12] found that political instability has a significant negative impact on economic growth in Pakistan. The authors suggest that political instability can reduce investor confidence, discourage foreign investment, and create an uncertain environment that hinders economic growth. According to [13] that the co-movement pattern between stock market, crude oil market and bitcoin market was effected by the pandemic and the political unrest. [14] also explain that the stock market index of one economy effected by the crisis and other factors in the neighborhood or international market. However, like the other consequences political instability also effect the local market as well as its spread to international market.

A study by [15] found that political instability has a negative impact on fiscal performance in Pakistan. The authors suggest that political instability can lead to government instability, policy uncertainty, and disruptions in the implementation of fiscal policies, which can negatively impact economic performance. A study by [16] found that political instability has a significant negative impact on foreign direct investment (FDI) in Pakistan. The authors suggest that political instability can create an uncertain environment that discourages foreign investors from investing in the country. According to [17] that the stock market including the other assets such as bitcoin and the energy derivates effected through different events and the crisis, and events may be the demographic or internal factors of the political unrest. Moreover, [18] also define the consequences of the political instability within the country that effect the bitcoin price and the energy commodities in Ukraine.

Overall, these studies suggest that there is a relationship between political instability and stock market performance evidence around the globe. Therefore, political instability led to uncertainty and reduced investor confidence, which can negatively impact stock market returns and increase volatility. However, the relationship between political instability and stock market performance is complex and influenced by other macroeconomic factors as well. Previous literature suggests that the relationship between political instability and economic performance may vary between emerging and developed economies. In emerging economies, political instability has been found to have a particularly negative impact on economic performance. Similarly, a study by [19] found that political instability had a significant negative effect on economic growth in Nigeria. Therefore, a study by [20] found that political instability had a negative impact on economic performance in Pakistan. In contrast, the impact of political instability on economic performance in developed economies is less clear. Some studies suggest that political instability may have a relatively smaller impact on economic performance in developed economies due to their greater institutional stability and political resilience. However, study by [21] found that political instability had a smaller impact on economic growth in developed economies than in emerging economies. However, from these cited studies we extracted that there is also gap of the knowledge to discuss the problem in term of the latest time and in that country where the political instability trend is increasing with respect to time. [22] found that political instability had a negative impact on economic growth in European Union countries and its impact varies with respect to time. On the ground of the previous literature, we developed the following hypothesis,

***H1*:** Political instability has a significant negative impact on the stock market performance.
***H2*:** Control of Corruption has a significant positive impact on the stock market performance.
***H3*:** There is a significant positive impact of Voice and accountability on stock market performance.
***H4*:** Government effectiveness has a significant positive impact on the stock market performance.
***H5***: Rules of law have a significant positive impact on the stock market performance.
***H6***: Regulatory quality has a significant positive impact of the Stock market performance.

## 3. Methods

### 3.1 Data description and sample size

This study covers Pakistan in which peoples of the economy faced the political instability from the last many decades that has the impact on their economic development. Pakistan is selected as a sample due to the increase in the political instability from last two decades. Moreover, another reason of the selection of the Pakistan as a sample Pakistan has experienced significant political instability since its inception in 1947. The country has gone through numerous military coups, political assassinations, and changes in government, making it a compelling subject for studying the dynamics of political instability over time. To meet our objectives of the study, we used the 50 years data from 1971 to 2021 on an annual basis. These economy data is selected due to the involvement of the foreign affairs in the country’s political situation. Some external factors have control over the political background. The data of the MSCI indices of Pakistan are collected from the DataStream data base. The WGI indicators data is collected from the world bank data portal (https://info.worldbank.org/governance/wgi/). The Conceptual model developed on the basis of the previous theory and literature are given in the Fig 1. Moreover, the Table 1 shows the variable measurement.

**Fig 1:** Conceptual framework.

**Table 1:** Variables measurement.

*Variable Name*		*Sign*		*Measurement*	*Reference*
Political Stability	PS		Estimate of governance (ranges from approximately -2.5 (weak) to 2.5 (strong) governance performance)		Worlds governance indicators by world
Control of corruption	CC		Estimate of governance (ranges from approximately -2.5 (weak) to 2.5 (strong) governance performance)		Worlds governance indicators by world https://info.worldbank.org/governance/wgi/
Voice and accountability	VA		Estimate of governance (ranges from approximately -2.5 (weak) to 2.5 (strong) governance performance)		Worlds governance indicators by world https://info.worldbank.org/governance/wgi/
Government effectiveness	GE		Estimate of governance (ranges from approximately -2.5 (weak) to 2.5 (strong) governance performance)		Worlds governance indicators by world https://info.worldbank.org/governance/wgi/
Rules of Law	RL		Estimate of governance (ranges from approximately -2.5 (weak) to 2.5 (strong) governance performance)		Worlds governance indicators by world https://info.worldbank.org/governance/wgi/
Regulatory quality	RQ		Estimate of governance (ranges from approximately -2.5 (weak) to 2.5 (strong) governance performance)		Worlds governance indicators by world https://info.worldbank.org/governance/wgi/
Stock market performance	STK		Measured by MSCI index value		Jain, M., Sharma, G. D., & Srivastava, M. (2019)

### 3.2 Variables measurement

Econometric model of the study that used in the analysis are given,

$$STK_{\mathrm{it}}=\alpha_{0}+\beta_{1}PI_{\mathrm{it}}+\beta_{2}VA_{\mathrm{it}}+\beta_{3}CC_{\mathrm{it}}+\beta_{4}RQ_{\mathrm{it}}+\beta_{5}RL_{\mathrm{it}}+\beta_{6}GE_{\mathrm{it}}+\varepsilon_{\mathrm{it}}$$

It is very essential the checking of the accuracy of the results of the stock market performance that leads to financial performance of the economy through the Robust analysis. Robust analysis is also useful for the accuracy of the result by one type measures and that’s why we used the GDP as the measure of the financial performance that corelate with the Stock market performance of any economy. The Robustness analysis equation are given below,

$$GDP_{\mathrm{it}}=\alpha_{0}+\beta_{1}PI_{\mathrm{it}}+\beta_{2}VA_{\mathrm{it}}+\beta_{3}CC_{\mathrm{it}}+\beta_{4}RQ_{\mathrm{it}}+\beta_{5}RL_{\mathrm{it}}+\beta_{6}GE_{\mathrm{it}}+\varepsilon_{\mathrm{it}}$$

The Ordinary Least Squares (OLS) method is a popular statistical technique used in business analysis to estimate the relationship between a dependent variable and one or more independent variables. OLS is commonly used in regression analysis to identify the strength and direction of the relationship between variables. In another study used OLS regression analysis to examine the relationship between ethical leadership and employee well-being [23]. Moreover, the OLS method has been widely used in business analysis to investigate various relationships and inform decision-making. Its versatility and ease of use have made it a popular technique among researchers and practitioners alike. Regression analysis is also a powerful tool for analyzing data and can be used to make predictions and forecast future trends. There have been numerous studies that have highlighted the usefulness of regression analysis in various fields, including finance, economics, and medicine. One recent study examined the relationship between economic growth and foreign direct investment (FDI) in the ASEAN region. The researchers used multiple regression analysis to analyze the data [24]. Another used regression analysis to examine the relationship between stock market returns and exchange rates in China [25]. In the field of medicine, a study used regression analysis to analyze data on patient satisfaction with healthcare services [26]. These studies demonstrate the usefulness of regression analysis in diagnosing the relationship between two or more variables in a range of fields. It allows researchers to identify significant relationships and make informed decisions based on data-driven insights. This study utilizes a quantitative methodology, analyzing time-series data on a key economic indicator, namely the Stock Market. To carry out this investigation, the study draws on data from the MSCI index and the Political Instability WGI indicators for Pakistan. The GMM method is used for robustness analysis. Generalized Method of Moments (GMM) is used for estimating parameters in econometric models and other statistical models. It is particularly useful when dealing with models that have endogenous variables and instruments to address issues related to omitted variable bias and measurement error. GMM is widely used in various fields, including economics, finance, and social sciences.

## 4. Findings and discussions

### 4.1 Descriptive statistics

Table 2 signifies descriptive statistics for our study for the data of Pakistan. The study model includes a total of 50observation for every variable. The table demonstrates that Corruption Control has a mean assessment of -0.937456 standard deviations of 0.13949 it is our independent variable. Whereas Government Effectiveness which is our independent variable has a mean of -0.619013and a standard deviation of 0.134657. In the same way, MCSI has a mean assessment of 2.6509and a standard deviation of 0.1542. Political stability has to mean assessment of -2.09038 and standard deviation of 0.550707. The rule of law has a mean assessment of -0.8172 and a standard deviation of 0.115192. Regularity Quality has a mean assessment of -0.6755 and a standard deviation of 0.123. Voice of Accountability has a mean assessment of -0.860523 and a standard deviation of -0.1736. Fig 2 shows the graphs of the value of the political stability and the other governance indicators.

**Fig 2:** Graph of the political stability and other governance indicators.

**Table 2:** Descriptive statistics.

	CC	GE	MSCI	PS	RL	RQ	VA
Mean	-0.937456	-0.619013	2.650959	-2.09038	-0.817292	-0.6755	-0.860523
Median	-0.89491	-0.624155	2.734322	-2.269401	-0.838977	-0.648122	-0.840511
Maximum	-0.777167	-0.380625	2.824144	-1.104805	-0.62529	-0.479762	-0.544719
Minimum	-1.22003	-0.82937	2.301197	-2.810035	-1.000389	-1.049112	-1.220254
Std. Dev.	0.13949	0.134657	0.154242	0.550707	0.115192	0.12387	0.173691

### 4.2 Correlation matrix

In our correlation matrix Table 3, CC and GE has the correlation value of 0.2740 which is less than the standard of 0.80. It means that there is not at all correlation between CC and GE. In the same way correlation matrix, CC and MSCI has the correlation value of 0.2689 which is less than the standard 0.80. It means that there is no correlation between CC and MSCI. Similarly, CC and PS have a correlation value of -0.1569 which is less than our standard 0.80. It means that there is no correlation between CC and PS. Now correlation matrix CC and RL Duality has the correlation value 0.2155 which is less than the standard 0.80. It means that there is not at all correlation between CC and RL. In our Correlation matrix, CC and RQ has a correlation value of 0.1309 which is less than the standard of 0.80. It means that there is not at all a correlation between the CC and RQ. In the same way in our correlation matrix, CC and VA have the correlation value of -0.0811 which is less than the standard of 0.80. It means that nearby is no correlation between CC and VA. Similarly, in our correlation matrix GE and MSCI has the correlation value of -0.4518 which is less than the standard of 0.80. It means that there is no correlation matrix among GE and MSCI. Our correlation of matrix RL and RQ has the correlation value of 0.4051 which is less than the standard of 0.80. It means that there is no correlation between RL and RQ. In the same way, RQ and VA have the correlation value of 0.6207 which is greater than standard, but it is the dependent variable, and the Scholar runs the reliant on variables RL, RQ AND VA separately so there is no impact on it. In our Correlation matrix, VA and VA have the correlation value is 01 in which both variables are the dependent variable.

**Table 3:** Correlation matrix.

	CC	GE	MSCI	PS	RL	RQ	VA
CC	1						
GE	0.274	1					
MSCI	0.2689	-0.4518	1				
PS	-0.1569	0.6969	-0.7114	1			
RL	0.2155	-0.0142	0.5401	-0.0203	1		
RQ	0.1309	-0.0883	0.3312	-0.3276	0.4051	1	
VA	-0.0811	-0.297	0.4183	-0.2668	0.6568	0.6207	1

### 4.3 Results and findings

The R-Square and Adjusted R value is 0.3540 and 0.3271, respectively indicating the about 32% effect is represented by the selected variable in the model and more other variable has impact but they does not included in the study and their probability is significant at 1% indicating the estimation fitness. In our results related to Pakistan in Table 4, Government effectiveness has significant at 5% level of significant, it means that Government effectiveness (GE) has positive impact on the stock market of Pakistan and also indicating that the 1 unit increase in the government effectiveness will rise in the 0.131749 in the stock market prices. Moreover, when the government has effective policies then there is growth in the financial markets leads to prosperity in Pakistan. Moreover, Political stability (PS) has significant at 1% and positive coefficient, it means that Political stability play very important role in stock market performance. When the political stability rises then increase in the 0.24 in the stock market indices of Pakistan. Similarly, in our results Rules of law (RL) and Voice and Accountability has significant positive impact on the stock market and it indicate that the 1 increase in the rules of law by the government then there should be 0.9191 increase in the stock market index of Pakistan. Moreover, it also indicated that when complete law and order is followed by the government then there is increase in the stock market due to the investor confidence increases on the stock. However, voice and accountability findings is also significant, indicating that 1 increase in the voice and accountability or freedom of choice leads to rise in the stock market index by 0.1441.

**Table 4:** OLS results of Model 1 (MSCI as a dependent variable).

Variable	Coefficient	Std. Err.	t-Statistics	Prob.
CC	-0.049456	0.155621	-0.317799	0.7547
GE	0.131749	0.216931	0.607328	0.0522**
PS	0.242331	0.053816	-4.502907	0.0004***
RL	0.919192	0.214528	4.284712	0.0006***
RQ	-0.141447	0.187761	-0.753338	0.4622
VA	0.144166	0.167853	-0.858882	0.0031***
R-Square	0.3540			
Adjusted R	0.3271			
Probability	0.0000***			

Significant at 1%***, 5%**, and 10% * levels of significance.

### 4.4 Robustness analysis

The value of the R-Squared value of our model in Table 5 that is estimated is 0.499018 and has the p-value is 0.055381 that talks about the model fit. In our results on the Stock Market Performance taken as a proxy for the GDP then Control variables Has important positive impact on the Stock market performance at 1% level of the significant, it means that all the indicators of the world governance have positive impact on financial performance of the economy that hit the stock market performance. Our robust analysis result verifies the existing results of the MSCI indices taken as the proxy for the stock market performance leads to financial performance of the economy because the stock market of any economy is considering the barometer of the country that drives the economic activities.

**Table 5:** Robust results of Model 3 (GDP as a dependent variable)ok.

Variable	Coefficient	Std. Err.	t-Statistics	Prob.
CC	4.319590	1.710107	2.525918	0.0225**
GE	1.735094	2.383836	0.727858	0.0772*
PS	1.978942	0.591384	-3.346292	0.0041***
RL	12.99600	2.357429	5.512785	0.0000***
RQ	6.921578	2.063283	-3.354643	0.0040***
VA	0.078208	1.844517	0.042400	0.9667
R-Square	0.499018			
Adjusted R	0.471049			
Probability	0.055381***			

Significant at 1%***, 5%**, and 10% * levels of significance.

In Table 6, the J-statistics value and its probability falls under significant region indicating the model fitness. Our results of the robustness shows that there is improvement in the findings as compared from the OLS methods. Control of the corruption in the regression method results are not significant but in the GMM method its relationship with the stock market performance is significant that indicated 1 point increase in the control of corruption within the country leads to 0.1892 in stock price due to significant positive impact of the control of the corruption on the stock market. Moreover, regulatory quality findings is not significant but in the GMM findings their results shows the significant and positive indicating that the regulatory quality of the governance has increase the stock market index.

**Table 6:** Robustness analysis through GMM method.

Variable	Coefficient	Std. Err.	t-Statistics	Prob.
CC	0.189261	0.13817	-0.42190	0.0547**
GE	0.23410	0.18941	0.58290	0.0013***
PS	0.291687	0.03415	-3.45321	0.0000***
RL	0.784131	0.19254	2.34165	0.0000***
RQ	0.82710	0.16123	-1.65123	0.0000***
VA	0.24162	0.23981	-0.78531	0.0001***
J-Statistics	0.8771			
Probability	0.0000***			

Significant at 1%***, 5%**, and 10% * levels of significance.

### 4.5 Discussion

Our findings related to Pakistan demonstrate that Government effectiveness has a significant positive impact on the stock market of Pakistan at the 5% level of significance. This indicates that when the government implements effective policies, there is growth in the financial markets which leads to prosperity in Pakistan. There is a large body of literature exploring the relationship between government policies and stock market performance. Overall, the literature suggests that government policies can have a significant impact on the stock market, both positively and negatively. Some policies that are generally considered to be positive for the stock market include those that promote economic growth, such as investment in infrastructure and tax cuts for businesses. Other policies that can have a positive impact on the market include those that promote stability and predictability, such as a clear and consistent regulatory environment.

On the other hand, policies that are viewed as negative for the stock market include those that create uncertainty and volatility, such as sudden changes in regulations or trade policies. Government policies that increase taxes or impose new regulations on businesses can also have a negative impact on the stock market. It is important to note that the relationship between government policies and the stock market can be complex and nuanced, and there are many factors that can influence stock market performance. Other factors that can affect the stock market include economic indicators such as interest rates, inflation, and GDP growth, as well as global events such as natural disasters or geopolitical conflicts. Overall, while there is evidence to suggest that government policies can have an impact on the stock market, the relationship is not always straightforward and is subject to a variety of other influences.

Additionally, our results show that Political stability plays a crucial role in the stock market performance, with a significant positive coefficient at the 1% level of significance. This means that when political stability rises, there is a 0.24 increase in the stock market indices of Pakistan. In this way, our results are supported by different previous literature. There have been several studies examining the relationship between political stability and the stock market in Pakistan. One study conducted by [27] found that political stability has a positive impact on the stock market and in this way our findings are consisted with [27] findings. The study used quarterly data from 1997 to 2016 and employed the autoregressive distributed lag (ARDL) model to estimate the long-run and short-run relationship between political stability and the stock market. The results of the study showed that political stability has a significant positive impact on the stock market in both the short and long run. Our results are similar with the findings of [28] that investigated the impact of political instability on the stock market in Pakistan using monthly data from 2000 to 2016. The study used the ARDL approach to examine the long-run and short-run relationship between political instability and the stock market. The results indicated that political instability has a negative and significant impact on the stock market in Pakistan in both the short and long run. Similarly, a study by [29] examined the relationship between political instability and stock market returns in Pakistan using monthly data from 1997 to 2011. The study employed the Granger causality test and found a bi-directional causality between political instability and stock market returns, suggesting that political instability and stock market returns have a mutually reinforcing relationship. Overall, the previous study literature suggests that political stability is an important factor influencing the stock market performance in Pakistan. While some studies have found a positive impact of political stability on the stock market, others have reported a negative impact. There are several instances where political instability has led to a decline in Pakistan’s stock market. For example, in 2018, the country’s stock market witnessed a significant decline due to political uncertainty surrounding the general election.

Similarly, our findings reveal that Rules of law (RL) and Voice and Accountability also have a significant positive impact on the stock market, suggesting that when the government follows complete law and order, investor confidence increases, leading to an increase in the stock market. Research has suggested that good governance, as measured by the rule of law (RL) and voice and accountability (VA), may have a positive impact on stock market performance. Our results are similar to the study that found RL and VA were positively associated with stock market returns in a sample of emerging market economies [30]. The authors suggest that RL and VA may create a stable and predictable business environment, which can encourage investment and promote economic growth. Another study analyzed data from 31 emerging markets and developing economies and found that stronger RL was associated with higher stock market returns and lower volatility [31] and in this way our study shows similar findings. Moreover, [31] also suggest that RL helps to promote transparency, accountability, and investor protection, which can increase investor confidence and encourage investment. A more recent study analyzed data from 63 countries and found a positive relationship between RL, VA, and stock market performance. [32] that validate our findings in this study through a justification. They suggest that RL and VA may lead to improved corporate governance, which can increase investor confidence and improve stock market performance. It is important to note that the relationship between RL, VA, and stock market performance may be influenced by a variety of other factors, such as economic conditions, political stability, and global events.

## 5. Conclusions and implementation

The economy can be greatly affected by political instability, which is usually reflected in the MSCI index value. This article highlights the negative impact of political instability on the economy and its reflection on the value of the MSCI index. Investors may pull their money out of the country’s stock market, leading to a decline in the value of the MSCI index and stocks. The MSCI value index measures the performance of stocks in Pakistan using market capitalization data from Pakistan stock exchange. It provides investors with information on the overall performance of the region’s economy and its risk and potential return for investment. The findings of the research indicate a strong correlation between political instability and a decline in the MSCI value index in Pakistan particularly in emerging economies. This has been supported by previous studies which have shown that when political instability rises, the MSCI value index decreases.

It is important to recognize that the MSCI index value serves as only one indicator of the economic growth and decline of Pakistan. Other factors, such as investment, exports, and government policies, also significantly impact the regions’ economic performance. Therefore, this study recommends that future research explore the relationship between government policy, investment, exports, and the economic performance of Pakistan. Our study advocated the implications for the investors, government and the policy makers. Based on the findings of this study, governments take measures to address political instability and establish a stable political environment. This can be achieved through policies that promote political stability, like constitutional reforms, and by addressing the root causes of political instability, such as poverty and inequality. By using the findings of the research, the governments and the policy makers can improve transparency and accountability in the political system to boost investor confidence. The policy makers in Pakistan can compare their political condition compared to other emerging countries, through they can balanced their resources of the current accounts and control some unrest factors. Therefore, it is important for governments and policymakers to address political instability and take measures to promote stability and security. This can include implementing policies that promote good governance, transparency, and accountability, as well as addressing the underlying causes of political instability, such as economic inequality and social unrest. Investors may also take steps to mitigate the impact of political instability on their investments. Investors make the diversification of their portfolios, investing in sectors that are less affected by political instability, and closely monitoring political developments and events. In addition, companies may take steps to address political instability and its impact on their operations and performance. This can include implementing risk management strategies, such as hedging against political risk and diversifying their operations geographically, as well as engaging with governments and stakeholders to promote stability and security. Future research should be conducted on the political instability effects on the social as well as intellectual capital of the economy. Moreover, another study should discuss the future topic by conducting the study on other emerging economies and compare it with developed economy world governance.

## Supporting information

S1 Data (XLSX)

S2 Data (XLSX)
